RETRACTED

# Expression and role of ABIN1 in sepsis: *In vitro* and *in vivo* studies

**DOI:** 10.1515/med-2021-0008

**Published:** 2020-12-04

**Authors:** Haolan Li, Aichen Sun, Taocheng Meng, Yan Zhu

**Affiliations:** Department of Infectious Diseases, Zaozhuang Municipal Hospital, Zaozhuang, 277102, China; Department of Orthopaedics, Zaozhuang Municipal Hospital, No. 47 Longtou Road, Zaozhuang, Shandong 277102, China; Department of ICU, Zaozhuang Municipal Hospital, Zaozhuang 277102, China

**Keywords:** ABIN1, inflammation, macrophages, sepsis

## Abstract

In this research, we attempted to explain the effect and the related molecular mechanisms of ABIN1 in lipopolysaccharide (LPS)-induced septic mice or RAW264.7 macrophages. LPS was adopted to treat RAW264.7 macrophages for 4 h, and the levels of inflammatory factors were assessed by ELISA. Besides, ABIN1 expression was measured by quantitative reverse transcription polymerase chain reaction. Apparently, LPS enhanced immunoreaction, suggested by increased expression of IL-1β, tumor necrosis factor (TNF)-α, and IL-6. ABIN1 levels were obviously reduced compared to the control. Furthermore, we evaluated the roles of ABIN1-plasmid in immunoreaction and nuclear factor-κB (NF-κB) pathway. We found that ABIN1-plasmid significantly reduced the expression of IL-1β, TNF-α, and IL-6 in LPS-treated cells and inhibited NF-κB pathway activation. Meanwhile, a septic mouse mode was conducted to validate the role of ABIN1 in inflammatory response and organ damage *in vivo*. These data suggested that ABIN1-plasmid significantly inhibited the secretion of inflammatory cytokines and Cr, BUN, AST, and ALT levels in the serum of LPS-stimulated mice compared to LPS + control-plasmid group, reflecting the relieved inflammation and organ injury. In summary, the present findings indicated that ABIN1 alleviated sepsis by repressing inflammatory response through NF-κB signaling pathway, emphasizing the potential value of ABIN1 as therapeutic strategy for sepsis.

## 1 Introduction

Sepsis is defined as severe systemic inflammatory reaction, it contributes to multiple tissues and organ dysfunction, and the process is intricate [1,2]. Currently, the morbidity and mortality of sepsis remain high around the world. Although great advancements have been made to decrease the mortality, there are still rare effectively apply in sepsis treatment. Certainly, understanding the mechanism of sepsis will be a benefit for the therapy of sepsis.

Macrophages, an important part of innate immune system, are related to various diseases and play a vital role in sepsis by regulating immune responses and inflammatory factors secretion, such as tumor necrosis factor (TNF)-α, IL-10, and IFN-g [3,4]. Recent research has indicated that excessive production of inflammatory cytokines was observed during sepsis [5,6]. Therefore, controlling macrophages activity and preventing abnormal activation were potentially powerful strategies for sepsis treatment. Lipopolysaccharide (LPS) is widely used to explore inflammation *in vivo* and *in vitro* models, where it stimulates many inflammatory factors [7]. For example, Araya et al. revealed that LPS induced TNF-α, IL-1β, IL-6, and PGE2 secretion in the whole blood of patients with Type 1 diabetes mellitus [8].

RETRACTED

Accumulating evidences have shown that numerous factors induce inflammation, including nuclear factor-κB (NF-κB) [9]. NF-κB pathway, a regulator in inflammation process, is associated with many diseases. NF-κB family includes five members, such as p65 (RelA), RelB, c-Rel, p50/105 (NF-κB1), and p52/p100 (NF-vB2), which exist in unstimulated cells as homo- or heterodimers bound to inhibitory κB (IκB) family proteins [10]. The released p65/p50 NF-κB dimer is transferred from the cytoplasm to the nucleus, binds to specific DNA sequences, and promotes the transcription of target genes [11,12]. In the classical pathway, NF-κB activation triggers the production of pro-inflammatory cytokines and NO [13,14]. Researches have revealed that classic NF-κB pathway inhibition can prevent the production of pro-inflammatory cytokines [15,16]. ABIN1, a homologue of ABIN proteins, was defined as a suppressor of immune system and plays important roles in immunity regulation as well as tissue homeostasis [17]. ABINs have been described as three different proteins (ABIN-1, ABIN-2, and ABIN-3), which bind to the ubiquitin-edited NF-κB inhibitor protein A20, and show limited sequence homology [18,19]. Upregulation of ABINs inhibits the activation of NF-κB through TNF and several other stimuli [18]. Similar to A20, the expression of ABIN1 is also dependent on NF-κB, which suggests a potential role of the A20/ABIN complex in the negative feedback regulation of the activation of NF-κB [18,19]. Previous study suggests that upregulation of A20/ABIN1 leads to macrophage polarization during infection [20]. However, the roles of ABIN1 in the development of sepsis need to be further explored.

In this research, the enhanced inflammatory factors levels and decreased ABIN1 mRNA and protein expression were observed in LPS-treated macrophages. It was subsequently determined that ABIN1-plasmid significantly increased the levels of ABIN1 and suppressed the inflammatory cytokines compared to LPS treatment group. Furthermore, ABIN1-plasmid was indicated to depress the p-p65 levels and reduced the ratio of p-p65/p65. All the data above indicated that ABIN1-plasmid protects against the secretion of LPS-stimulated pro-inflammatory cytokines by inhibiting NF-κB signal activation in macrophages. Further study indicated the anti-inflammation and organ-protective effects of ABIN1-plasmid on *in vivo* model.

RETRACTED

In conclusion, our study provided novel evidence that ABIN1 is an important regulator and participated in the progression of sepsis by activating the NF-κB pathway.

## 2 Materials and methods

### 2.1 Animals

C57BL/6 mice (20–24 g) were purchased from the Model Animal Center of Shanghai and were adopted in this study at 6–8 weeks age. The mice were kept in a temperature- and humidity-controlled room with free-issue diet and drinking. All animal procedures were conducted referring to the National Institutes of Health Guide for the Care and Use of Laboratory Animals and were approved by the Institutional Animal Care and Use Committee (IACUC) of Zaozhuang Municipal Hospital.

### 2.2 Animal model

The mice were adapted to the standard condition for 2 weeks before experiment. Then we grouped the mice into the control and the sepsis group (*n* = 10 for each group). LPS (10 mg/kg; Santa Cruz, CA) was adopted to establish sepsis model, and the control group received normal saline. At 24 h after LPS treatment following the last injection, ABIN1-plasmid (80 mg/kg/day) or control-plasmid (80 mg/kg/day) was injected by tail intravenous injection for three consecutive days. After that, the mice were anesthetized using pentobarbital (30 mg/kg, intraperitoneal injection), and the blood was subsequently harvested and centrifuged to extract serum for histopathological evaluation at 24 h after LPS treatment as detailed earlier. The mice health and behavior were observed every 2 days. During our experiment, no mice died. Throughout the whole experiment, we did our best to alleviate the pain of the mice, and experiments were ended when the mice lost more than 15% of their body weight.

### 2.3 Cell culture and LPS stimulation

The RAW264.7 macrophage was cultivated in DMEM (Gibco, USA), including 10% FBS and 1% penicillin/streptomycin. Then macrophage was incubated in an incubator with 5% CO_2_. In this study, macrophage was treated with 1 μg/mL LPS for 4 h and harvested for further research.

### 2.4 Cytokines and organ injury markers’ detection

After LPS treatment for 24 h, blood was collected from each group, centrifuged (1,600 × *g*, 15 min), and the supernatant was gathered for analysis. IL-1β, IL-6, and TNF-α levels from serum were quantitatively detected using ELISA (BD biosciences). Serum ALT, AST, Cr, and BUN were measured to assess organ damage, referring to the manufacturer’s instructions.

RETRACTED

The expression levels of IL-1β, IL-6, and TNF-α in the cell supernatant were also detected using ELISA kits (Beyotime, Shanghai, China), according to the manufacturer’s protocols.

### 2.5 Cell transfection and reagents

Macrophage cells were planted into a 6-well plate and cultured for 24 h, with cell transfection performed when the cell density was up to 50–60%. For transfection, control-plasmid (cat no. sc-437275; Santa Cruz Biotechnology) or ABIN1-plasmid (cat no. sc-425441-ACT; Santa Cruz Biotechnology) was transfected into macrophages using Lipofectamine^®^ 2000 reagent (Invitrogen, Carlsbad, CA), referring the manufacturer’s protocol. After that, RAW 264.7 macrophages were induced by LPS for 4 h and the transfection efficiency was conducted by quantitative reverse transcription polymerase chain reaction (qRT-PCR) and western blot analysis.

### 2.6 qRT-PCR

TRIzol reagent (Thermo Fisher Scientific, MA) was adopted to isolate total RNA from serum and macrophages, following the manufacturer’s protocol. PrimeScript™ RT reagent kit (TaKaRa) was adopted to synthesize cDNAs. Then we detect ABIN1 levels by real-time PCR system, referring to the manufacturer’s protocol. GAPDH was regarded as control. Primer sequences were obtained from Sangon Biological and listed as follows:

GAPDH-forward, 5′-AAGGTTCGGAGTCAACGGA-3′;

reverse, 5′-TTAAAAGCAGCCCTGGTGA-3′;

ABIN1-forward, 5′-GTGTTCCGATGTGGCTCT-3′;

reverse, 5′-ACCCACTCCTCCTTGGC-3′.

Amplification conditions were as follows: after 5 min denaturation at 95°C, 40 cycles were conducted including 95°C for 15 s, 60°C for 1 min, 55°C for 1 min, and final step at 72°C for 10 min. The target genes expression was assessed by 2^−ΔΔCq^ method.

### 2.7 Western blot analysis

Cells’ proteins were extracted by RIPA lysis buffer (Beyotime) and each sample was subjected to 10% SDS–PAGE. Then they were transferred onto PVDF membranes (Owl Scientific) and the membranes were incubated with blocking solution for 1 h. Anti-GAPDH (1:1,000; Abcam), anti-ABIN1 (1:1,000; Abcam), anti-p65 (1:1,000; Abcam), and anti-p-p65 (1:1,000; Abcam) were applied as primary antibodies. After washing with PBST for four times, membranes were incubated with secondary antibody for 1 h. The proteins were quantified using ECL detection reagent (Pierce Biotechnology).

### 2.8 Statistical analysis

SPSS 20.0 statistical software (IBM Corp.) was adopted to analyze the statistics. All the results were represented as mean ± SD from three independent experiments. Student’s *t*-test and ANOVA followed by Student–Newman–Keuls tests were applied for evaluating differences between the groups. We considered statistically significant as *p* < 0.05.

RETRACTED

## 3 Results

### 3.1 LPS treatment reduced ABIN1 levels and decreased inflammatory factors’ secretion in RAW264.7 macrophages

As is well acknowledged that sepsis is related to immunoreaction. First, macrophages were stimulated by LPS for 4 h, and the IL-1β, IL-6, and TNF-α levels were evaluated using ELISA to assess the immunoreaction. We observed that expression of inflammatory factors was obviously higher in LPS-treated group than that in control (Figure 1a–c). Moreover, we analyze the ABIN1 levels by qRT-PCR and western blot assays, respectively. Our data showed that ABIN1 was downregulated in LPS-stimulated macrophages (Figure 1d and e). These data indicated that ABIN1 may be involved in sepsis progression.

**Figure 1:** Expression of ABIN1 was suppressed and inflammatory cytokines were enhanced in LPS-induced macrophages. Macrophages were stimulated by 1 μg/mL LPS for 4 h. (a) TNF-α, (b) IL-1β, and (c) IL-6 levels in RAW264.7 macrophages. (d) ABIN1 mRNA and (e) protein expression in macrophages were assessed by qRT-PCR and western blot assay, respectively. **p < 0.01 vs control.

### 3.2 ABIN1-plasmid suppressed the expression of inflammatory factors in LPS-stimulated macrophages

The above results that we obtained indicate that ABIN1 participated in the development of sepsis. Then we explored the potential pathogenesis of ABIN1 in LPS-induced macrophages. Macrophages were transfected with control-plasmid or ABIN1-plasmid for 48 h, followed by 4 h LPS treatment. As shown in Figure 2a, ABIN1-plasmid prominently enhanced the ABIN1 mRNA (Figure 2a) and protein levels (Figure 2b) in macrophages, compared with control. Multiple relative researches indicated that excessive inflammatory response often appeared during the progression of sepsis; thus we detected the inflammatory cytokines by ELISA in different groups. We observed upregulation of inflammatory factors in LPS-treated macrophages. On the contrary, compared to LPS group, secretion of LPS-inducible cytokines was remarkably inhibited after ABIN1-plasmid treatment (Figure 2c–e). The aforementioned further revealed that ABIN1 regulated the inflammatory reaction in macrophages.

**Figure 2:** ABIN1-plasmid reversed the effects of LPS on inflammatory factors in macrophages. (a) mRNA and (b) protein levels of ABIN1 in macrophages after ABIN1-plasmid transfection. After transfection with control-plasmid or ABIN1-plasmid, the levels of (c) TNF-α, (d) IL-1β, and (e) IL-6 in different groups were determined. ^&&^ *p* < 0.01 vs control-plasmid; **p < 0.01 vs control, and ^##^ *p* < 0.01 vs LPS + control-plasmid.

### 3.3 ABIN1-plasmid inhibited NF-κB pathway activation in LPS-stimulated macrophages

Western blot assay was adopted to evaluate the related protein expression. Results from Figure 3a showed that LPS increased the p-p65 levels compared with control, whereas the effects were reversed in ABIN1-plasmid + LPS group. Moreover, the same variation trend of p-p65/p65 was observed in different groups, and we found that p-p65/p65 were enhanced after LPS treatment and decreased by ABIN1-plasmid (Figure 3b). The aforementioned suggested that ABIN1 exerted an important role in inflammatory development by activating NF-κB pathway *in vitro.*

RETRACTED

**Figure 3:** ABIN1-plasmid suppressed LPS-stimulated NF-κB activation in macrophages. Control-plasmid or ABIN1-plasmid was transfected into macrophages for 48 h, followed by LPS treatment. (a) Western blot analysis was adopted to evaluate p-p65 and p65 expression in four groups (control, LPS, LPS + control-plasmid, and LPS + ABIN1-plasmid). (b) Ratio of p-p65/p65. **p < 0.01 vs control, and ^##^ *p* < 0.01 vs LPS + control-plasmid.

### 3.4 ABIN1-plasmid protects against the effects of LPS on liver injury in septic mice

To assess the effects of ABIN1 on immunoreaction and LPS-stimulated liver injury *in vivo*, LPS was applied to conduct sepsis model followed by control-plasmid or ABIN1-plasmid stimulation. qRT-PCR was conducted to measure ABIN mRNA levels in LPS-induced mice serum. The results indicated that ABIN1 mRNA was remarkably suppressed in LPS-treated mice serum compared to control group (Figure 4a). However, the effects of LPS on ABIN1 mRNA were alleviated by ABIN1-plasmid (Figure 4a). Furthermore, ELISA assay was applied to assess the release of inflammatory factors in mice serum in different groups (control, LPS, LPS + control-plasmid, and LPS + ABIN1-plasmid). As shown in Figure 4b–d, we found increased inflammatory factor levels in the LPS-induced mice serum. However, the secretion of inflammatory factors was remarkably inhibited in the serum of LPS + ABIN1-plasmid-treated mice compared with LPS + control-plasmid group (Figure 4b–d).

**Figure 4:** LPS affected the inflammatory factors’ secretion and liver damage. (a) qRT-PCR analysis was carried out to evaluate ABIN1 expression. Secretion of (b) TNF-α, (c) IL-1β, and (d) IL-6 in serum were verified using ELISA assay in control and LPS groups. (e) Serum Cr, (f) BUN, (g) ALT, and (h) AST levels were determined in control and LPS groups. **p < 0.01 vs control, and ^##^ *p* < 0.01 vs LPS + control-plasmid.

To further verify the positive impact of ABIN1-plasmid on LPS-stimulated liver injury *in vivo*, ELISA assay was carried out to analyze the liver damage alterations. Our results suggested that the levels of serum kidney and liver injury markers (Cr, BUN, ALT, and AST) were increased after LPS treatment compared to control (Figure 4e–h). These effects of kidney and liver injury markers on LPS-induced mice were significantly reduced in ABIN1-plasmid combination treatment group (Figure 4e–h). The above data showed that ABIN1 prevented the inflammatory response progression in septic mice.

RETRACTED

## 4 Discussion

Sepsis remains the main cause of morbidity and mortality in clinic worldwide, mainly caused by immune response [21,22,23]. Various reports have highlighted that immune cells are involved in sepsis, including macrophage. Macrophage has been reported to mediate inflammation-related diseases by releasing inflammatory factors [24,25]. Moreover, it is reported that LPS is often used to stimulate macrophages in *in vivo* or *in vitro* models. Excessive accumulation of inflammatory factors is the main cause of organ dysfunction syndrome in sepsis [26]. Based on these, in our research, we explored deeply that the effects of macrophages on sepsis are essential to cure sepsis. First, we provided evidence that the secretion of inflammatory cytokines was promoted in LPS-induced macrophages. In accordance with our findings, Bian et al. reported that LPS significantly enhanced the production of inflammatory factors in macrophages [27].

ABIN1 is an A20-binding protein, which functions as an inhibitor in NF-κB pathway [28]. Various investigations have revealed that ABIN1 was participated in many diseases. For example, Zhou et al. found that ABIN1 controls beta protein activation and protects from inflammatory disease [29]. In addition, Korte et al. showed that ABIN1 determines glomerulonephritis severity by activating intrinsic glomerular inflammation [30]. However, whether ABIN1 is involved in the formation of sepsis and the mechanism of it remain unclear. Based on the aforementioned research, this study aimed to elaborate the role of ABIN1 in sepsis. qRT-PCR and western blot analysis were conducted to evaluate ABIN1 mRNA and protein levels in RAW264.7 macrophages treated with or without LPS. In support of this result, previous studies have confirmed that ABIN1 was significantly downregulated in LPS-treated RAW264.7 macrophages. Therefore, we imagined that upregulation of ABIN1 expression might exert anti-inflammatory functions in sepsis. We further transfected control-plasmid or ABIN1-plasmid into RAW 264.7 macrophages for 48 h, and then the cells were treated with 1 μg/mL LPS for further 4 h. We found that ABIN1-plasmid significantly increased ABIN1 levels and alleviated the secretion of inflammatory factors in LPS-induced macrophages. Taking these data into consideration, our results indicated that ABIN1 regulated immunoreaction in sepsis.

RETRACTED

As we all know, the inflammatory response is resulted from many signaling pathways, among which NF-κB pathway is the major regulator to the inflammatory genes [31]. In addition, several reports have revealed that suppression of NF-κB promoted LPS-stimulated sepsis [32]. We subsequently detected the expression of NF-κB-related proteins by western blot assay. Our findings showed that the protein expression of p-p65 and p-p65/p65 ratio was enhanced after LPS treatment, whereas these changes were reduced by ABIN1-plasmid. The above results revealed that ABIN1 regulated immunoreaction by inhibiting the NF-κB pathway activation *in vitro.*

LPS is a kind of endotoxin in combination with receptors in multiple vectors, including macrophage [33]. Thus, LPS injection is often used to conduct an animal model of sepsis. Based on *in vitro* functions of ABIN1 in regulating immune response in macrophages, we further tried to research the influence of ABIN1 on immune response in LPS-induced sepsis model *in vivo*. After 72 h of LPS injection, we detected ABIN1 mRNA and inflammatory factors’ release by qRT-PCR and ELISA, respectively. We found lower ABIN1 mRNA levels and higher inflammatory factors production in the serum of mice in LPS group than that in the control group. However, these changes were reversed in LPS + ABIN1-plasmid group. During sepsis development, organ dysfunction usually occurs in systems [34,35]. In this study, we determined the Cr, BUN, ALT, and AST levels in mice serum, which represent the kidney and liver dysfunction. The kidney and liver dysfunction marker levels were enhanced in LPS-treated mice, whereas these results were attenuated after ABIN1-plasmid treatment. We provided evidence that ABIN1-plasmid repressed the inflammatory response in septic mouse.

Studies have shown that overexpression of ABINs inhibits the activation of NF-κB through TNF and several other stimuli [18,36]. It has recently been shown that ABINs contain an ubiquitin-binding domain, which is essential for their NF-κB inhibitory activity [37,38]. In this case, it was proposed that ABINs act as adaptors between ubiquitinated proteins and other regulatory proteins [37,38]. However, in this study, the regulation mechanism of the inhibition of ABIN1 on NF-κB signaling pathway is unclear, which needed further investigation. In addition, whether the baseline levels of Cr, BUN, ALT, and AST affect the anti-inflammatory effects of ABIN1-plasmid remain unclear. This was a limitation of the current study. We will explore this more in-depth in future research.

Taken together, this report verified the anti-inflammatory effects of ABIN1-plasmid on both *in vitro* and *in vivo* inflammatory models. For all we know, it was the first time to elucidate the mechanism of ABIN1 in sepsis, and the mechanism involved in the regulation of inflammatory response in sepsis of ABIN1 was shown in Supplementary Figure S1. Our research provided a promising therapeutic strategy for sepsis treatment.
